The article "Assessment of the Impact of Higher Education on Environmental Quality in BRICS Economies Based on Sustainable Development Pathways" was retracted in 2023. Reasons: signs of a paper mill; suspected computer-generated content; unreliable results or conclusions; concerns about the data.

# Assessment of the Impact of Higher Education on Environmental Quality in BRICS Economies Based on Sustainable Development Pathways

**DOI:** 10.1155/2022/6447763

**Published:** 2022-09-22

**Authors:** Miao Guo

**Affiliations:** ^1^Northeast Normal University, Changchun, Jilin 130000, China; ^2^Changchun University, Changchun, Jilin 130022, China

## Abstract

From the perspective of ecological environmental protection, higher education can not only train a large number of professionals dedicated to environmental protection for the construction of environmental quality, but more importantly, it can promote the improvement of the quality of ecological civilization in the whole society, so as to achieve the effect of indirectly improving environmental quality. BRICS economies, as the most important economies in the world, have an impact on the development of the world in many aspects. However, under the guidance of the concept of sustainable development, whether the environmental quality of BRICS economies meets the standards has also become the focus of scholars. Starting from the sustainable development path, this paper summarizes the model of environmental education in BRICS national higher education. At the same time, through the establishment of the BRICS environmental quality assessment system, the environmental quality of the BRICS countries after the implementation of environmental education was assessed based on the content of the sustainable development system. This paper performs matrix operations on the weight values of the indicators at all levels and the membership vector to obtain a 4 × 4 matrix, that is, the evaluation result *Q* of each indicator is [0.050, 0.200, 0.113, 0,011], which proves that the evaluation results in this paper are basically reasonable. It can be seen that in terms of forest coverage and environmental protection areas, environmental education in higher education has the deepest impact on Russia. In terms of carbon emissions, South Africa benefits the most from environmental education in higher education, so each country should take corresponding actions according to different environmental assessment results.

## 1. Introduction

As the external space for the development of a region, its quality determines the development of other aspects of the region, especially the economy. If the environmental quality is maintained well, it can provide a basis for economic development, and at the same time attract foreign investment and introduce people to live a virtuous circle in the region. However, if the environmental quality is not good, it will not only cost a lot of financial expenditures for external improvement but also will be difficult to maintain in the subsequent development, resulting in a rebound, which is likely to form a vicious circle and damage other aspects of development. Since the concept of sustainable development and green development was put forward, environmental quality has been continuously evaluated and studied in various forms because it is closely related to economic development. School is an important place for environmental quality education, and various types of schools play a major role in the process of environmental quality education. Young people are the key groups of environmental quality, and colleges and higher education should be the main positions for the implementation of environmental quality education. The construction of a country with green mountains, clean water, blue sky, and fresh air requires not only high-level planners and scientific and technological talents who are passionate about environmental protection but also the majority of ordinary workers with high ecological civilization quality. However, the cultivation and shaping of these talents needed by the society basically depends on education, especially the environmental quality education. As several major economies that make great economic contributions to the world, the BRICS countries' development path is more worthy of in-depth discussion, so it is of practical significance to study the impact of higher education on environmental quality.

The article "Assessment of the Impact of Higher Education on Environmental Quality in BRICS Economies Based on Sustainable Development Pathways" was retracted in 2023. Reasons: signs of a paper mill; suspected computer-generated content; unreliable results or conclusions; concerns about the data.

Environmental quality is closely related to everyone's quality of life and has always been a hot topic of research by scholars. Abdouli examined the impact of environmental quality and capital stock on economic growth in 17 MENA countries. By the systematic generalized moments panel data method, his findings show that economic growth in MENA countries negatively responds to environmental quality [1]. His research provided ideas for us to avoid environmental degradation, but there is still a lack of countermeasures to improve environmental quality. Abid proposed through research that there is a monotonically increasing relationship between CO_2_ emissions and GDP in the Middle East, Africa, and the European Union [2]. His research is instructive on the balance between environmental quality and economic development, but the experimental procedures are not rigorous enough. Raju et al. used geospatial technology to assess environmental quality by taking thermal power plants as an example [3]. Although his research has a guiding role in improving environmental quality, the scope of his research is too narrow. Liu et al. proposed that although rapid urbanization leads to the deterioration of urban environmental quality, it has limited impact on the spatial pattern and driving factors of urban environmental quality in mountainous cities in China [4]. Although their research has obtained valid results, it also has the problem that the research area is too narrow. Paramati et al. studied the impact of tourism on economic growth and environmental CO_2_ emissions in Eastern and Western European Union countries by incorporating FDI and trade into the production and CO_2_ emission functions [5]. Their research shows that tourism adversely affects the environmental quality of Eastern Europe, but there is no valid validation of the same adaptation in other regions.

The article "Assessment of the Impact of Higher Education on Environmental Quality in BRICS Economies Based on Sustainable Development Pathways" was retracted in 2023. Reasons: signs of a paper mill; suspected computer-generated content; unreliable results or conclusions; concerns about the data.

As an important path for human survival and development, sustainable development path has been widely used in different object research centers since it was proposed. Wu and Zhang introduced environmental quality and nonrenewable resources as endogenous factors and constructed a sustainable growth model with dual constraints of resources and environment [6]. Although his research is extensive, the derivation process is too complicated. Taking India as an example, Srikanth proposed to develop innovative strategies to clean up the country's coal sector while strengthening the integration of renewable energy into the national grid from a sustainable path [7]. His research is exemplary for developing countries, but not in all regions. Syangbo introduced the integration of sustainable development paths and organic farming practices from an educational perspective [8]. His research is very helpful for the education of sustainable development path, but the research is still relatively simple and not deep enough. Pietrzak et al. analyzed the quality of the entrepreneurial environment at the regional level in Poland under the framework of sustainable development paths [9]. Their research takes Poland as an example, which has a unique perspective, but lacks specific guidance and suggestions, and is not practical.

From the perspective of sustainable development path, this paper evaluates the environmental quality of BRICS countries after the implementation of environmental education in higher education. The innovation of this paper mainly lies in the diversification and multiangle of the environmental assessment of the BRICS countries, and it is further subdivided from the three perspectives of forest coverage, climate conditions, and environmental protection areas. The situation and data of each country are visually presented and compared, which makes the analysis of the article more accurate and objective.

## 2. Methods for Assessing the Impact of Higher Education on the BRICS Environmental Quality

### 2.1. Sustainable Development Path

The concept of sustainable development comprehends social development as the quality of human life and the overall optimization of the natural and human environment. The sustainable development path is fundamentally different from the traditional development path. In contrast, sustainable development needs to first solve the universal problem of the nonsustainable problems of contemporary economic and social development, so that development can be transferred to a benign track, and the ecological and social costs of economic and social development can be reduced to a minimum [10]. It essentially reflects the concept of developing and implementing the concept of ecological civilization.

The article "Assessment of the Impact of Higher Education on Environmental Quality in BRICS Economies Based on Sustainable Development Pathways" was retracted in 2023. Reasons: signs of a paper mill; suspected computer-generated content; unreliable results or conclusions; concerns about the data.

The basic concepts of sustainable development concept are its premise is development, its goal is to increase human well-being and improve the quality of human life, and it focuses on the harmony and unity of the economy, society, population, environment, and resources. The sustainable development path is to use the conditions and opportunities of contemporary people to create an environment that can continue to develop, leaving a harmonious and green space for future generations. Rather than impair or jeopardize the ability and condition of future generations to meet their needs, future generations should also enjoy reasonable and equal opportunities for development. In the pursuit of human rights of development, we must always maintain a harmonious and mutually beneficial relationship with nature, organically combine economic development and ecological sustainable development, and achieve it in a harmonious and natural way. The development and utilization of the environment, resources, and energy must be within the control and carrying capacity of the ecosystem, instead of the traditional way of increasing investment, increasing consumption and sacrificing the environment, which balances production's demand for resources with the environment's availability of resources.

Specifically, the connotation of sustainable development can be understood from another perspective into three aspects: fairness, sustainability, and commonality [11]. The connotation of fairness refers to the fairness of contemporary people, which means that sustainable development should meet the basic needs of all people and give the world fair distribution and fair development rights. At the same time, when distributing the resources of the present generation fairly, the resource utilization of future generations should also be considered, and the limited resources should be distributed fairly [12]. The connotation of sustainability means that sustainable development should not destroy the ability of environmental regeneration, and human economic and social activities should ensure that the environment can bear the living. For example, sustainable development should not destroy the natural ecosystems that support life on Earth: the atmosphere, water, soil, organisms, etc. The connotation of commonality means that all human beings should be united to maintain sustainable development. Because sustainable development is not the goal of individual regions nor the fate of individual groups, it requires the joint efforts of all countries and regions. Based on the above description, a framework diagram of the sustainable development path can be drawn, as shown in Figure 1.

The article "Assessment of the Impact of Higher Education on Environmental Quality in BRICS Economies Based on Sustainable Development Pathways" was retracted in 2023. Reasons: signs of a paper mill; suspected computer-generated content; unreliable results or conclusions; concerns about the data.

### 2.2. Environmental Education Models in Higher Education in BRICS Countries

Under the guidance of the sustainable development path, as a formal national education, higher education can make use of its various advantages in environmental quality education, give full play to its positive role in cultivating talents needed by society, and improve the civilized quality of young people. With the guidance of the concept of sustainable development, the BRICS countries also attach equal importance to environmental protection in higher education. Colleges and universities in various countries have combined relevant teaching content, popularized ecological environment knowledge, and incorporated advanced and necessary content of various environmental quality educations into their teaching plans, so that young people can receive good environmental quality education. Therefore, it will be invested in the construction of sustainable development in the future [13]. Through literature review and data research, this section investigates the higher education policies of five BRICS countries and summarizes the environmental education methods of higher education in each BRICS country, mainly including the following:

*Classroom Teaching*. Classroom teaching is not only the most basic way of higher education but also the place where the largest amount of information is imparted. In the classroom, teachers can have the opportunity to instruct students how to help students carry out environmental quality transformation from the perspective of sustainable development. Teachers of various subjects use classroom penetration to organically integrate the specific goals of ecological civilization education into the process of subject classroom teaching, strengthen their awareness of ecological protection, and improve their ecological civilization quality and behavioral ability while learning relevant knowledge [14]. From the perspective of higher education, universities in BRICS countries not only provide ecological environment majors but also nonecological environment majors with corresponding education on ecological civilization and environmental protection. In BRICS countries, for students majoring in ecological environment and other related majors, environmental protection education continuously improves educational methods and means to further improve educational effects [15].

The article "Assessment of the Impact of Higher Education on Environmental Quality in BRICS Economies Based on Sustainable Development Pathways" was retracted in 2023. Reasons: signs of a paper mill; suspected computer-generated content; unreliable results or conclusions; concerns about the data.

*Second Classroom*. The second class refers to the nonclassroom but also the form of classroom teaching effect, such as lectures and special reports. Relevant topics and reports can make full use of modern educational technology (such as multimedia, projector, and network) to mobilize the enthusiasm and pertinence of students to participate in the activities without destroying the academic and authoritativeness of the subject content and prepare for the activities in advance. In BRICS countries, the second classroom of higher education can be seen everywhere. Lectures to promote environmental protection are often held among students. Report activities advocating sustainable development are also emerging one after another, so as to improve students' awareness of environmental protection [16].

*Campus Culture Construction*. In BRICS countries, this kind of educational significance is no less than simply instilling the awareness of protecting the environment and saving resources in students. At the same time, this form can also have a positive impact on students' awareness of ecological civilization in a subtle way [17]. In addition, in BRICS countries, when schools carry out popularization of ecological environment knowledge, more students are introduced to understand, and the concept of sustainable development and environmental quality protection is further expanded [18]. The construction of campus culture helps to build not only the school culture but also the culture of national ecological protection.

*Extracurricular Practical Activities*. In higher education in BRICS countries, in addition to the above forms, practical activities are also one of the good ways of environmental quality education. In these countries, it is common for colleges and universities to jointly carry out public welfare activities oriented to the society, with the theme of saving resources and planting trees, and guide people to cooperate with nonprofit environmental protection organizations. Jointly carry out socially oriented ecological civilization education and practical activities with the theme of saving resources and rejecting pollution [19]. Carry out various missionary activities for the society. Taking college students' ecological and environmental protection associations as an important carrier to carry out various publicity and education activities also promotes the improvement of environmental quality invisibly [20]. It can not only deepen students' understanding of the concept of ecological environmental protection and exercise their social practice ability but also play an important role in promoting the direct transmission of the concept of ecological civilization in the whole society.  Figure 2 shows the protection model of environmental quality in higher education in BRICS.

The article "Assessment of the Impact of Higher Education on Environmental Quality in BRICS Economies Based on Sustainable Development Pathways" was retracted in 2023. Reasons: signs of a paper mill; suspected computer-generated content; unreliable results or conclusions; concerns about the data.

### 2.3. Construction of BRICS Environmental Quality Assessment System

This section will use the fuzzy evaluation model to build an evaluation system for the environmental quality of BRIC countries. The fuzzy comprehensive evaluation is based on fuzzy mathematics, which was first proposed by experts in cybernetics in the United States. After that, it has experienced rapid development and is now used in many aspects, including industry, environment, and agriculture. Fuzzy comprehensive evaluation can effectively reduce the subjectivity of evaluation results, evaluate some objective fuzzy phenomena more accurately, determine the boundaries of evaluation objects from multiple aspects, and improve evaluation accuracy [21].

*The Determination of the Evaluation Index Set*U

(1) $$\begin{array}{c} U=\left\{u_{1},u_{2},u_{3},\cdots ,u_{n}\right\}, \end{array}$$

where u_*i*_(*i* = 1, 2, ⋯, *N*) represents the evaluation index, and *N* is the number of evaluation indexes in the same layer.

*Determination and Standardization of Evaluation Grades*

(2) $$\begin{array}{c} V=\left\{V_{1},V_{2},V_{3},\cdots ,V_{n}\right\}, \end{array}$$

where *V*_*j*_(*j* = 1, 2, ⋯, *n*) represents the comment level, and *n* is the number of levels. The rating scale can be a quantitative numerical value or a qualitative description.

*Determination of Membership Vector*

If the single-factor evaluation of the *i*-th evaluation factor u_*i*_ is V_j_

(3) $$\begin{array}{c} R_{\text{i}}=\left(r_{i1}.r_{i2},r_{i3}\cdots ,r_{ij}\right),i=1,2,\cdots ,N;j=1,2,\cdots ,n, \end{array}$$

where r_*ij*_ represents the degree of membership of factor u_*i*_ in v_*j*_, and 0 ≤ r_*ij*_ ≤ 1. By analogy, the membership degree of n elements is a matrix of N rows and n columns. In this paper, the membership function is used to calculate the membership of each element.

(4) $$\begin{array}{c} {\text{y}}_{i}=\beta_{o}\left(u_{i},v_{i}\right)+\sum \begin{array}{c} p\\ k=1 \end{array}\beta_{k}\left(u_{i},v_{i}\right)x_{ik}+\varepsilon_{i} \end{array}$$

In the formula, y_*i*_ represents the dependent variable value of sampling point *i*; *β*_o_ is the intercept, (u_*i*_, *v*_*i*_) is the scalar value of *i*; *β*_o_(*u*_*i*_, *v*_*i*_) is the constant term of *i*. *β*_k_(*u*_*i*_, *v*_*i*_)**is** the coefficient of the *k*-th independent variable of *i*, and x_*ik*_ is the *k*-th independent variable of sample *i*; *ε*_i_ is the random error term of i.

The article "Assessment of the Impact of Higher Education on Environmental Quality in BRICS Economies Based on Sustainable Development Pathways" was retracted in 2023. Reasons: signs of a paper mill; suspected computer-generated content; unreliable results or conclusions; concerns about the data.

*Multilevel Comprehensive Evaluation*

According to the evaluation principle of the maximum membership degree, the evaluation level of each index is determined, and the final evaluation result is obtained [22].

(5) $$\begin{array}{c} Q=R_{i}*B_{i} \end{array}$$

Among them, *Q* is the ecological environment quality of the evaluation unit, *R*_*i*_ represents the membership degree matrix of the first-level evaluation index, and *B*_*i*_ represents the combined weight of the first-level evaluation index.

## 3. Environmental Quality Experimental Design and Data Sources

This section discusses the data sources of the experiment and the design of the relevant analysis process. The data for the analysis of the experimental results in this article are from the data of the BRICS National Bureau of Statistics and the national statistical yearbooks of various countries [23]. The data sources can be obtained from the official websites of various countries and official announcements. BRICS has cooperated with many parties since its establishment in 2011. The data in this section on the impact of higher education on environmental quality are from 2017 to 2021. Since its establishment in 2011, the universities in the five BRICS countries have completed the planning of environmental protection education and the arrangement of environmental quality courses. After 2017, it was five years after the first batch of higher education on environmental quality ended. From the analysis of environmental quality in the past five years, it can be concluded that the effect of higher education on environmental quality and the trend of BRICS national environmental development, the research path of this paper is sustainable development. Therefore, in the results section, corresponding statistical analysis will be carried out on the data and performance of each country's environmental quality from the perspective of sustainable development.

## 4. Results Analysis

### 4.1. Deconstruction of Forest Cover Results

Forest cover has a significant impact on a country's environmental quality, and countries and regions with high forest cover mean that places can deal with carbon emissions more easily. At the same time, the forest area determines the size of the ecosystem. As a complex and huge ecosystem, the forest can provide shelter for animals and it can provide a growing environment for plant diversity, which further affects human activities [24]. The analysis of forest coverage in this section is carried out from three perspectives, namely, forest area, proportion of forest coverage, and plant diversity. This section analyzes the data of the “Global Forest Resources Assessment” in recent years to obtain the forest vegetation coverage data of BRICS countries and statistics the results as shown in Figure 3.

The article "Assessment of the Impact of Higher Education on Environmental Quality in BRICS Economies Based on Sustainable Development Pathways" was retracted in 2023. Reasons: signs of a paper mill; suspected computer-generated content; unreliable results or conclusions; concerns about the data.

From Figures 3(a) and 3(b), it can be seen that from 2017 to 2021, the trend of forest coverage in the five BRICS countries has basically maintained a similar level. But Brazil has a downward trend, especially from 499.53 million hectares to 498.07 million hectares from 2019 to 2020. The 1 million hectares lost is not only related to the development of forest resources in Brazil to promote urbanization but also part of it is related to the fires in the Amazon forest. Among these five countries, Russia not only has the largest forest area, but also maintains the highest growth trend, with a total increase of 300,000 hectares from 2017 to 2021. The geographical environment of Russia, which is vast and sparsely populated, provides advantages for forest growth and area expansion [25]. As for the forest coverage rate of the rest of the countries, China has a relatively prominent performance. The forest area is large, but the land area is also large, so the forest coverage rate is not the highest.

As can be seen from Figure 3(c), in terms of forest vegetation diversity, according to the International Assessment Rules for Forest Plant Diversity, China has the highest average proportion of forest vegetation diversity in BRICS countries, and within 5 years, it has basically maintained a normalized high diversity rate. Among them, South Africa has the lowest diversity, which is not only related to the low forest coverage rate in South Africa (the average area is 1.7 million hectares) but also has a great relationship with the geographical location of the country.

### 4.2. Deconstruction of the Results of the Climate Environment

Climate factors, including temperature, precipitation, sunshine hours, and carbon emissions have an important impact on the regional environment. Different climate types correspond to different vegetation types, and the ecological conditions formed by different vegetation types are different [26]. Therefore, climate plays an important role in the ecological environment quality of BRICS countries. In this study, because each country has a very large area and spans a very wide range of latitudes and longitudes, it is difficult to summarize with one temperature level or climate type. Therefore, the climate factors are divided into two indicators: carbon emissions and temperature changes.  Table 1 shows the variation of annual mean temperature in BRICS countries.

The article "Assessment of the Impact of Higher Education on Environmental Quality in BRICS Economies Based on Sustainable Development Pathways" was retracted in 2023. Reasons: signs of a paper mill; suspected computer-generated content; unreliable results or conclusions; concerns about the data.

Combining with the temperature analysis in Table 1, it can be concluded that although the temperature changes of BRICS countries are not very different within their respective countries, the average temperature of some countries is slightly abnormal. There are many factors that affect temperature. Although the most important one is the climate factor, because each country has many dimensions and different climates, the change in average temperature can fairly show the results of temperature change. In order to further analyze the climate and environment of BRICS countries, through the arrangement of global carbon emission data, the article obtained the statistical results of total carbon emission and per capita carbon emission growth rate as shown in Figure 4.

From the carbon emission results in Figure 4, it can be seen that after planning environmental quality courses in higher education, the best carbon emission control in BRICS countries is South Africa, with an average per capita carbon emission of only 10 kg per year, far lower than other countries, while China and Russia have the highest carbon emissions. Among them, China's carbon emissions are higher than Russia's, and the per capita annual carbon emissions can reach about 10,000 kilograms. This is also related to China being the most populous country in the world. The large population base and high energy use rate lead to China's carbon emissions reaching the highest among the five countries. China's carbon emissions have a downward trend, which is also related to the “carbon neutrality” and “carbon peaking” policies implemented by China.

### 4.3. Deconstruction of Environmental Protection Zone Results

In addition to forest coverage, environmental protection areas are also one of the criteria for measuring environmental quality. In this section, the statistics on environmental protection areas mainly include the number of environmental protection areas and the proportion of biodiversity. The number of environmental protection areas also includes natural forest parks, wildlife reserves and national parks and other protection areas. The criteria for determining biodiversity and the proportion of data come from the “International Handbook of Common Biological Conservation”. After statistics, the statistical results in Figure 5 can be obtained.

From the statistical results in Figure 5, it can be seen that among the BRICS countries, the construction and maintenance of environmental protection zones is the best in Russia. The protected areas in Russia not only show an increasing trend year by year but also the highest number of protected areas reaches more than 100 in a year. In 2019, the number of protected areas reached 11,864, while Brazil and China were slightly behind in the number of protected areas. Among them, the number of protected areas in China shows a decreasing trend every year, from 2,750 to 480. Although Brazil has increased from a low of 320 to 400, the total number is still the lowest. Therefore, China and Brazil need more investment in the construction of environmental protection zones.

The article "Assessment of the Impact of Higher Education on Environmental Quality in BRICS Economies Based on Sustainable Development Pathways" was retracted in 2023. Reasons: signs of a paper mill; suspected computer-generated content; unreliable results or conclusions; concerns about the data.

### 4.4. Comprehensive Assessment of Ecological Environment Quality

After analyzing the results of various environmental factors in the above content, this section takes the Fuzzy Comprehensive Appraisal (FCE) method introduced in Section 2 as the basic method for evaluation. Analytic Hierarchy Process (AHP) and Coefficient of Variation (CPA) were used to determine the comprehensive weight of each indicator, and then comprehensively evaluate the environmental quality of BRICS countries. The fuzzy evaluation method performs fuzzy operations on each index in the study area, which largely avoids the influence of human factors on the evaluation results, and the evaluation accuracy is high.

*Analytic Hierarchy Process (AHP) to Determine the Weight*. First, the weight of the evaluation index of the evaluation unit is calculated by the Analytic Hierarchy Process (AHP). Firstly, the matrix of each single factor index is constructed, and its consistency ratio is calculated. Because the consistency ratio is CR < 0.10, it means that the constructed matrix between each index can achieve satisfactory results, and the ranking and consistency ratio of the total level can be calculated continuously. Next, the total ranking and inspection of the hierarchy are calculated, as shown in Table 2.

It can be seen from Table 2 that in the calculation of the total hierarchical ranking, the CR value is 0.056 < 0.10, indicating that the matrix results constructed by the total hierarchical ranking can be used to determine the weight of each index and finally calculate the weight value of each single element to the target layer.

*The Coefficient of Variation Method (CPA) Determines the Weights*. According to the formula given in Section 2, the index weight based on CPA is calculated, and the objective weight value of each index of the evaluation unit is obtained. Using the linear combination method, by comprehensively calculating the weight values determined by APH and CPA, the comprehensive weight of each index of the evaluation unit is obtained, as shown in Table 3.

As shown in Table 3, according to the comprehensive weight value analysis, among the first-level evaluation indicators, the natural environment index has the largest weight, and the environmental protection area index has the smallest weight, which are 0.550 and 0.094, respectively. It reflects that the regional forest coverage rate has the greatest contribution to the regional ecological environment quality, while the impact degree of the environmental protection area is relatively low.

The article "Assessment of the Impact of Higher Education on Environmental Quality in BRICS Economies Based on Sustainable Development Pathways" was retracted in 2023. Reasons: signs of a paper mill; suspected computer-generated content; unreliable results or conclusions; concerns about the data.

*Fuzzy Comprehensive Evaluation*. Before the calculation of the fuzzy comprehensive evaluation model, it is necessary to determine which level each index belongs to, that is, the calculation of the membership degree of the evaluation index. Firstly, based on the quantitative value (usually the mean) of each secondary index in the middle, the trapezoidal distribution algorithm is used to calculate the membership degree of each secondary index. That is, the membership degree value of each single factor. According to the matrix operation method, perform matrix operation on the weight values of the indicators at all levels and the membership vector to obtain a 4 × 4 matrix, that is, the evaluation results of each indicator in the secondary indicators, as shown in Table 4 and Formula (6).

(6) $$\begin{array}{c} Q=R_{i}*B_{i}=\left[0.050\;0.200\;0.113\;0.011\right]. \end{array}$$

*Verification of Evaluation Results*. Due to the lack of field verification work, this study mainly refers to the existing literature and expert opinions to verify the evaluation results. First, studies have shown that after environmental protection courses are planned into higher education, among BRIC countries, Russia has the best ecological environment quality. However, Russia is only doing well in forest coverage and environmental protection areas, but its carbon emissions are among the highest among the five countries. As a result of comprehensive environmental quality, Brazil has the lowest comprehensive quality and basically has no advantages except for the relatively large proportion of forest coverage. The other three countries, China, India, and South Africa, have their own advantages and disadvantages, but the overall results are all at the medium quality level [27]. Compared with the analysis in this paper, combined with the results obtained by the expert scoring method and calculation, it can be said that the environmental quality evaluation results of this BRIC economy are basically reasonable.

## 5. Conclusion

As the emerging economies of the world, the BRICS countries have brought great influence and changes that cannot be underestimated. In addition to the growth of the economy under the influence of the BRICS countries, the world environment is also affected by the development activities of the BRICS countries. This article starts from the path of sustainable development and summarizes the environmental education of higher education in BRICS countries. Then, an environmental quality assessment system is constructed based on the comprehensive fuzzy evaluation method. In the conclusion analysis, the environmental quality of the BRICS countries is analyzed from the three perspectives of forest coverage, climate environment and environmental protection area, and finally the fuzzy comprehensive evaluation is carried out. The analysis results of the article show that higher education has had different environmental impacts on different countries since the arrangement of environmental education. In terms of forest coverage, Russia is the most affected and therefore has the highest forest coverage. At the same time, Russia has also done the best in environmental protection zones, and among the five countries in terms of carbon emissions, South Africa has performed the best. Although the article evaluates the environmental quality from different perspectives, due to the limited space, there is still a lot of detailed analysis and specific process descriptions in the research methods and experimental demonstrations, which is also the shortcoming of the article. In the future, people could look forward to conducting research based on more scientific methods and making contributions to the research on education and environmental protection.

The article "Assessment of the Impact of Higher Education on Environmental Quality in BRICS Economies Based on Sustainable Development Pathways" was retracted in 2023. Reasons: signs of a paper mill; suspected computer-generated content; unreliable results or conclusions; concerns about the data.

## Figures and Tables

**Figure 1:** Framework of sustainable development pathways.

**Figure 2:** Environmental quality protection model for higher education in BRICS.

**Figure 3:** BRICS national forest cover statistics results.

**Figure 4:** BRICS carbon emissions statistics.

**Figure 5:** Statistical results of BRICS environmental protection areas.

**Table 1:** Annual mean temperature change in BRICS countries.

	2017	2018	2019	2020	2021
Brazil	30.520	31.471	32.456	30.347	30.120
Russia	27.312	28.236	27.112	29.469	28.450
India	31.154	33.784	32.236	30.580	31.360
China	29.360	30.145	29.145	31.364	30.140
South Africa	28.874	27.324	30.013	28.457	29.214

**Table 2:** Hierarchical total ranking and inspection.

	Natural environment	Climate environment	Soil environment	Hydrological environment	W
Natural environment	1.000	3.000	5.000	3.000	0.499
Climate environment	0.333	1.000	6.000	2.000	0.282
Protection environment	0.200	0.167	1.000	0.500	0.073
Hydrological environment	0.333	0.500	2.000	1.000	0.146
	Target layer consistency ratio CR: 0.056; weight to target layer: 1.000				

**Table 3:** Composite weight values.

Evaluation target	First-level evaluation index	Value	Secondary evaluation index	Value
BRICS eco-environmental quality assessment	Forest cover rate	0.424	Forest area	0.200
			Coverage percentage	0.224
	Water resources	0.004	Freshwater resources	0.001
			Total water use	0.001
	Climate environment	0.354	Carbon dioxide emissions	0.232
			Temperature change rate	0.122
	Protected area	0.210	Number of protected areas	0.210
			Biodiversity as a percentage of protected area	0.008

The article "Assessment of the Impact of Higher Education on Environmental Quality in BRICS Economies Based on Sustainable Development Pathways" was retracted in 2023. Reasons: signs of a paper mill; suspected computer-generated content; unreliable results or conclusions; concerns about the data.

**Table 4:** Membership matrix of the first-level evaluation layer.

Evaluation factors	Good	Generally	Poor	Very poor
Natural environment	0.039	0.340	0.169	≤ 0.001
Climate environment	0.155	0.017	0.012	≤ 0.001
Protected environment	≤ 0.001	0.057	0.085	0.030
Hydrological environment	≤ 0.001	≤ 0.001	0.031	0.064

## Data Availability

The data used to support the findings of this study are available from the corresponding author upon request.
